# Phytotherapeutic Approach in the Management of Cisplatin Induced Vomiting; Neurochemical Considerations in Pigeon Vomit Model

**DOI:** 10.1155/2022/3914408

**Published:** 2022-09-13

**Authors:** Ihsan Ullah, Fazal Subhan, Muhammad Shahid, Nisar Ahmad, Rehmat Shah, Javaid Alam, Ikram Ul Haq, Rahim Ullah, Muhammad Ayaz, H. C. Ananda Murthy

**Affiliations:** ^1^Department of Pharmacy, University of Swabi, Swabi, Pakistan; ^2^Department of Pharmacy, Institute of Integrative Biosciences, CECOS University of IT and Emerging Sciences, Peshawar, KP, Pakistan; ^3^Department of Pharmacy, University of Peshawar, Peshawar, Pakistan; ^4^Department of Pharmacy, Islamia College of Pharmacy, Sialkot, Pakistan; ^5^Pharmacist, Health Department, Khyber Pakhtunkhwa, Pakistan; ^6^Drug and Herbal Research Center, Faculty of Pharmacy, University Kebangsan, Malaysia; ^7^National Institute of Health, Islamabad, Pakistan; ^8^Sarhad University of Science and Information Technology, Peshawar, Pakistan; ^9^Department of Pharmacy, Faculty of Biological Sciences, University of Malakand, Chakdara, 18000 Dir (L), KP, Pakistan; ^10^Department of Applied Chemistry, School of Applied Natural Science, Adama Science and Technology University, P O Box 1888, Adama, Ethiopia; ^11^Department of Prosthodontics, Saveetha Dental College & Hospital, Saveetha Institute of Medical and Technical Science (SIMATS), Saveetha University, Chennai 600 077, Tamil Nadu, India

## Abstract

Cisplatin induced vomiting involves multiple mechanisms in its genesis and a single antiemetic agent do not cover both the phases (acute & delayed) of vomiting in clinics; necessitating the use of antiemetics in combination. *Cannabis sativa* and other selected plants have ethnopharmacological significance in relieving emesis. The aim of the present study was to investigate the intrinsic antiemetic profile of *Cannabis sativa* (*CS*), *Bacopa monniera (BM,* family *Scrophulariaceae)*, and *Zingiber officinale* (*ZO*, family *Zingiberaceae*) in combinations against vomiting induced by highly emetogenic anticancer drug-cisplatin in pigeons. We have analysed the neurotransmitters which trigger the vomiting response centrally and peripherally. Electrochemical detector (ECD) was used for the quantification of neurotransmitters and their respective metabolites by high performance liquid chromatography in the brain stem (BS) and area postrema (AP) while peripherally in the small intestine. Cisplatin (7 mg/kg i.v.) induced reliable vomiting throughout the observation period (24 hrs). *CS*-HexFr (10 mg) + *BM*-MetFr (10 mg)–Combination 1, *BM*-ButFr (5 mg) + *ZO*-ActFr (25 mg)–Combination 2, *ZO*-ActFr (25 mg) + *CS*-HexFr (10 mg)–Combination 3, and *CS*-HexFr (10 mg) + *BM*-ButFr (5 mg)–Combination 4; provided ~30% (30 ± 1.1), 70% (12 ± 0.4; *P* < 0.01), 60% (19 ± 0.2; *P* < 0.05) and 90% (05 ± 0.1; *P* < 0.001) protection, respectively, against cisplatin induced vomiting as compared to cisplatin control. Standard MCP (30 mg) provided ~50% (23 ± 0.3) protection (*P* > 0.05). *CS* Hexane fraction (10 mg/kg), *BM* methanolic (10 mg/kg) and bacoside rich *n*-butanol fraction (5 mg/kg) and *ZO* acetone fraction (25 mg/kg) alone provided ~62%, 36%, 71%, and 44% protection, respectively, as compared to cisplatin control. The most effective and synergistic combination 4 was found to reduce 5HT and 5HIAA (P < 0.05–0.001) in all the brain areas area postrema (AP)+brain stem (BS) and intestine at the 3^rd^ hour of cisplatin administration. In continuation, at the 18^th^ of cisplatin administration reduction in dopamine (*P* < 0.001) in the AP and 5HT in the brain stem and intestine (*P* < 0.001) was observed. The said combination did not change the neurotransmitters basal levels and their respective metabolites any significantly. In conclusion, all the tested combinations offered protection against cisplatin induced vomiting to variable degrees, where combination 4 provided enhanced attenuation by antiserotonergic mechanism at the 3^rd^ hour while a blended antidopaminergic and antiserotonergic mechanism at the 18^th^ hour after cisplatin administration.

## 1. Introduction

Nausea and vomiting are the two important adverse effects faced by the patients undergoing cancer chemotherapy [1, 2]. These adverse effects may often result in noncompliance to the chemotherapy but it may result to the refusal of patients to undergo emetogenic chemotherapy cycles. It is known that the cancer is second in the United States which resulted in more deaths; and the studies advocate the increase in the number of cancer patients and, more importantly, breast, lungs, head and neck, colorectal, and stomach carcinomas [3–5].

The emetogenecity of antineoplastics varies and that is why they are also classified based on its emetogenic propensity. The high emetogenic class contains all the platinum analogues including cisplatin. Cisplatin has the unique aspect that induces vomiting in two phases; the first phase which stays up to 24 hours is known as acute phase while the phase after 24 hours is called delayed phase and it is believed today that it remains up to 7 days after the initiation of chemotherapy cycle. Mechanistically, the vomiting caused by cisplatin is multifactorial with respect to acute and delayed phases. The acute phase is triggered by serotonin; the primary neurotransmitter to be considered while neuropeptide “Substance P” is the mediator for delayed phase [6, 7]. Keeping in view the aforementioned mediators to trigger the vomiting response, the pharmacotherapy also varies in the management of this biphasic vomiting response. For the management of acute phase serotonin receptor blockers e.g. Ondansetron etc. are proved beneficial while the same has shown no significant control over the delayed phase of vomiting; being controlled by neurokinin 1 receptor antagonists (Apprepitant) in combination with dexamethasone. In clinical setups, the combination of antiemetics is used to control both the phases of vomiting induced by cisplatin by following the international guidelines, but still this is a clinical challenge, as the considerable proportion of patients undergoing cancer chemotherapy faces the problem of vomiting [8, 9] making it a need for a time to look for new antiemetic having a broad spectrum so it has the capability to control both the phases of vomiting.

The natural plants and the phytochemicals isolated from them are proved to be very important for ailing community and also provide structural templates for the new compounds to be developed [10–15]. The drugs like Quinine etc. have their source from plants and have still significance in the management of various diseases [16–22]. The scientific community is still involving in the isolation and characterization of active phytochemicals against various pathologies [23–25]. Recently, the standardization of extracts/fractions/isolates is getting much more attention to identify the active moiety responsible for the therapeutic response [26–30]. Keeping in view the biphasic vomiting response and the multimechanisms behind the two phases established the use of antiemetics in combination and provides the platform to search for a cost effective combination of herbal origin which may provide good control over the acute and delayed phases of vomiting in clinics. The current study is focusing on *Bacopa monniera* (*BM*), *Cannabis sativa* (*CS*), and *Zingiber officinale* (*ZO*) to see their impact on cisplatin induced vomiting either alone or in combination in the pigeon emesis model. Pigeon emesis model is good for preliminary screening of chemical entities/compounds/extracts/fractions for the antiemetic potential and has been used by the scientific community for the said purpose. Pigeon demonstrates a robust and very clear vomiting response as compared to *Suncus murinus* to almost all the emetogenics.

The literature is rich enough to advocate the antiemetic effect of *Cannabis sativa* and *Zingiber officinale* as antiemetic, while the antiemetic activity of *Bacopa monniera* is reported by our laboratory for the first time. The major chemical moiety of Cannabis extract i.e. *Δ*^9^-tetrahydocannabinal (*Δ*^9^-THC) has been shown to be antiemetic and also shown promising results in clinics [31, 32]. Furthermore, the *cannabis* preparations have shown superior antiemetic activity as compared to Dopamine receptor blockers [33]. The identification of endocannabinoids and cannabinoid receptors [34, 35] revolutionized the research in cannabinoids for the two decades.

*Zingiber officinale* is well known for its use as spice and flavouring agent and also been used for the treatment for vomiting and anorexia [36]. Gingirol is reported as the active component responsible for its activities along with some other moieties as well [36, 37]. Sharma and his coworkers have reported the antiemetic activity of ginger against cisplatin induced vomiting in dogs [38] and against cyclophosphamide induced vomiting in the *Suncus murinus* [39].

*Bacopa monniera* is well known for its significance in the management of memory impairments [40] and cognitive disorders [41]. The literature is indicating bacosides as the major and important chemical constituent responsible for its activities. The plant extracts are standardized by the prompittayarat in 2007 [42] and our laboratory also did the HPLC fingerprinting of *bacopa* extracts [43] indicating the bacosides as major constituents. Our studies also provided evidences for the mechanisms behind the antiemetic activity of bacosides against cisplatin induced vomiting in pigeon. Based on the previous reports as its antidopaminergic aspect and our findings the bacoside rich fraction is included in the current study.

The antiemetic activity of *CS*, *ZO*, and *BM* is well investigated alone. Keeping in view the mechanistically multifactorial phenomenon associated with cisplatin induced vomiting, we hypothesize that the combinations of these safe and tolerable plant extracts may exhibit a broad spectrum antiemetic activity which may be helpful to cover all the phase of vomiting caused by cisplatin in clinics.

## 2. Materials and Methods

### 2.1. Animals

Pigeons of both gender (male and female) and of all species (mix breed at the breeding facility of the Department) having weight in range of 250–350 g were used (*n* = 8). The light/dark cycle was kept as 12 hours and the food and water was available as usual. All the procedures to be done on experimental animals were first approved by the Ethical committee of the Department having the reference No 5/pharm and are according to the animal scientific procedure ACT, 1986 (UK).

### 2.2. Drugs and Chemicals

Methanol, acetonitrile, 1-octane suphonic acid (HPLC grade, Fisher scientific), EDTA, and sodium dihydrogen orthophosphate (Merck), Metoclopramide (GSK, Pakistan). The neurotransmitter standards (noradrenaline, dopamine, and serotonin) and their metabolites (DOPAC, 5HIAA, and HVA) were purchased from Acros Organics (Belgium). Cisplatin was gifted by the Korea United Pharm (Korea). Bacosides were gifted by the University of Mississippi USA. *N*-butanol, *n*-hexane, and acetone were from Haq Chemicals Pakistan.

### 2.3. Extraction and Fractionation of *Bacopa monniera*

*Bacopa monniera* (*BM*) was carefully collected near the locality of Quid-e-Azam University, Islamabad. A specimen was identified by taxonomist Prof. Dr. Muhammad Ibrar from University of Peshawar and the same was submitted to the Department of Botany herbarium for future reference (V # 7421). The plant required parts were collected, shade dried, and grinded. One kilogram plant material was first treated with *n*-hexane with solvent to crude drug ratio of 03 : 01 to remove all nonpolar components and then treated with acetone (01 : 0.9) for the purpose to remove fats and chlorophyll, then extracted using commercial grade methanol (03 : 0.7) using soxhelet apparatus and the yield was 28 grams. The product was further processed with *n*-butanol and the 1.6 grams of the fraction was obtained; which is the bacoside rich fraction [44, 45]. All the fractions were dissolved in distilled water for administration.

### 2.4. Extraction of *Cannabis sativa*

*Cannabis sativa* (*CS*) was collected at District Malakand KP, Pakistan at its flowering stage and later on authenticated by Prof. Dr. Muhammad Ibrar and a specimen was submitted to the Department herbarium with voucher number 8717. The required plant parts were collected, dried under shade, and then grinded. The grinded material was extracted as reported by our lab [46–48].

### 2.5. Extraction of *Zingiber officinale*

500 grams of the ginger rhizomes were purchased from local market at Mardan, Pakistan. A specimen was identified and the same is submitted to the herbarium with voucher number 20017–pup. The rhizomes were washed and crushed in a way to expose its inner part. Maceration procedure was used for extraction of active phytochemicals (yield 4.72%) [49].

### 2.6. Drug Formulation

The emetogenic drug cisplatin was dissolved in normal saline by gentle heating up to 60°C. The *n*-butanol (bacoside rich fraction) was dissolved in distilled water for administration. The *n*-hexane fraction of *CS* was dissolved in mixer of ethanol, emulsifier, and distilled water in ratio of 5: 5: 90, respectively [50, 51]. Ginger acetone fraction was dissolved in distilled water and sonicated for complete dissolution.

### 2.7. Drug Administration

Intramuscular route (Chest muscle) was used for administration of test extracts, standard, and vehicle, while intravenous route was used for administration of cisplatin. After cisplatin administration the animals were put back in confining cages and the behaviour was observed up to 24 hours. Standard antiemetic–metoclopramide, respective vehicles, and test extract combinations were administered 30 minutes before the administration of cisplatin. At the end of the experiment the body weight was noted to calculate body weight loss and the animals were euthanized.

### 2.8. Antiemetic Assay

Cisplatin was administered (7 mg/kg) and the behaviour of the animals was recoded for 24 hours [48, 52]. Food and water were available to the experimental animals as usual. The one vomiting episode was considered with or without the expulsion of stomach contents and the relaxed posture among the two episodes was considered the separation marker [53]. Further in the studies, cisplatin was used at the dose of 7 mg/kg to induce vomiting and to evaluate the antiemetic effects of various extracts alone or in combination.

### 2.9. Tissue Sampling for Neurotransmitters Analysis

The brain areas: (1). Area postrema and (2). Brain stem were collected at the end of experiment by following the Atlas [54, 55], which were later on processed for quantification of neurotransmitters and their metabolites. Intestinal samples were also collected 10 cm from the pylorus for HPLC-ECD analysis.

### 2.10. Determination of Neurotransmitters and Their Metabolites

The brain and intestinal samples were first cleared using cold saline and then homogenized in cold 0.2% perchloric acid at 5000 rpm using Teflon glass homogenizer, centrifuged at 12000 g/minute (4°C), filtered using 0.45 *μ* filter. High performance liquid chromatography was used along with electrochemical detector for quantification of neurotransmitter and their metabolites in brain areas and intestine as reported in our previous studies [56].

### 2.11. Statistical Analysis

One-way analysis of variance was applied as a tool for group comparison and Student *t*-test/tukey's multiple comparison test/Dunnett's test was used as post hoc tests by using GraphPad Prism (Version 8). *P* value less than 0.05 was considered as statistically significant. The animal which showed no vomiting response is excluded from latency calculations.

## 3. Results

### 3.1. Antiemetic Effect of *CS* Hexane Fraction (10 mg/kg), *BM* Methanolic (10 mg/kg), and Bacoside Rich *N*-Butanol Fraction (5 mg/kg), and *ZO* Acetone Fraction (25 mg/kg) Alone and in Combinations

To see for any possible synergistic combination among the selected plant extracts against cisplatin induced vomiting. The combinations tested were

1. *CS*-HexFr+*BM*-MetFr
2. *BM*-ButFr+*ZO*-ActFr
3. *ZO*-ActFr+*CS*-HexFr
4. *CS*-HexFr+*BM*-ButFr

Furthermore, all the fractions of *CS*, *BM*, and *ZO* most effective doses were also tested for their antiemetic effects alone as well.

The vomiting response of ~45 episodes with latency of ~66 minutes was recorded for cisplatin control, where all the animals showed reliable vomiting response up to the observation period (Table 1). Standard antiemetic metoclopramide suppressed the vomiting response to ~23 episodes (50%) and increased the latency up to 248 min (*P* > 0.05) as compared to cisplatin control. Combination 4 proved to be a synergistic combination as calculated by limpel equation [57] and it provided protection up to 89% (*P* < 0.001, Table 1) against the vomiting induced by cisplatin during the observation period. Combination 4 significantly increased the latency to first vomit as well (*P* < 0.01). Combination 2 reduced the vomiting episodes up to 12 (73%), while combination 3 provided up to 58% protection (~19 episodes) against cisplatin induced vomiting (*P* < 0.05, Table 1). Furthermore, Combination 1 also attenuated the vomiting response but nonsignificantly. Only combination 4 significantly (*P* < 0.01) increased the latency to first vomit while others failed to do so. The combination 4 provided enhanced protection and proved to be synergistic where it provided complete remission of vomiting response in one animal, although it attenuated the vomiting response to a maximum degree and increased the latency as well. Combination 4 in comparison to other combinations lowered the vomiting episodes but the difference was found to be statistically nonsignificant (Table 1, Figures 1–3). The most effective doses of the *CS* (10 mg/kg), *BM* methanolic (10 mg/kg), *BM n*-butanolic (5 mg/kg), and *ZO* (25 mg/kg) alone provided up to 62%, 36%, 71%, and 44% attenuation of vomiting as compared to cisplatin control (Table 1, Figures 1–3).

### 3.2. Effect of *CS* Hexane Fraction (10 mg/kg), *BM* Methanolic (10 mg/kg) and Bacoside Rich *N*-Butanol Fraction (5 mg/kg), and *ZO* Acetone Fraction (25 mg/kg) Alone and Combination 1, 2, 3, and 4 on Cisplatin-Induced Jerks and Weight Loss

Animals in control group (cisplatin treated) lost their body weight up to 15%, while the combination 1 and 3 showed the reduction in weight loss significantly (P <0.05–0.01, Table 1). In continuation, combination 2, 4, and standard metoclopramide failed to do so. No combination reduced the jerking episodes any significantly.

### 3.3. Effect of Standard MCP and Combination 4 on Basal Neurotransmitters Cum Metabolites in the Brain Areas and Intestine

Metoclopramide significantly reduced the concentration of 5 hydroxy indole acetic acid (5HIAA) in the area postrema and brain stem significantly (*P* < 0.05 and *P* < 0.001, respectively) as compared to basal level. Furthermore, the homovanillic acid (HVA) was also decreased significantly when compared with basal HVA concentration (Table 2). Combination 4 only reduced the concentration of 5HIAA in the brain stem as compared to basal level (*P* < 0.05, Table 2).

### 3.4. Effect of Metoclopramide and Combination 4 on Neurotransmitters Cum Metabolites in the Brain Areas and Intestine at 3^rd^ Hour of Cisplatin Treatment

The concentration of 5-hydroxy tryptamine was significantly increased (*P* < 0.001) in the brain stem and at the level of intestine as compared to vehicle treated, while in the area postrema a nonsignificant increase was observed (Table 3). Metoclopramide (30 mg/kg) did not changed the concentration of all the neurotransmitters and their metabolites in the brain areas and intestine but only reduced the concentration of 5-hydroxy tryptamine in the brain stem and intestine (*P* < 0.001) as compared to cisplatin control (Table 3). In continuation, metoclopramide also decreased the concentration of 5HIAA in the brain stem, area postrema, and intestine (*P* < 0.01–0.001, Table 3).

Combination 4 significantly (*P* <0.05–0.001) decreased the concentration of 5HT and its metabolite 5-hydroxy indole acetic acid (5HIAA) in the brain stem, area postrema, and intestine (Table 3). However, no significant effects were observed on the other neurotransmitters in the brain areas and intestine except dihydroxy pheny acetic acid (DOPAC) which was found significantly increased in intestine (*P* < 0.05, Table 3).

### 3.5. Effect of Metoclopramide or Combination 4 on Neurotransmitters Cum Metabolites in the Brain Areas and Intestine at 18^th^ Hour of Cisplatin Treatment

The concentration of neurotransmitter–Dopamine was significantly (*P* < 0.001) increased in the area postrema while a nonsignificant trend was observed in the brain stem and intestine (Table 4). 5HT concentrations were also noted to be increased in area postrema, brain stem, and intestine with significance of *P* < 0.01, *P* < 0.001, and *P* < 0.001, respectively, and did not affect the levels of others (DOPAC, HVA, 5HIAA, and NA) (Table 4). Metoclopramide decreased the dopamine surge significantly in area postrema (*P* < 0.001). In addition, the decrease in the concentration of 5HT was also observed in the area postrema (*P* < 0.01), brain stem (*P* < 0.001), and intestine (*P* < 0.001) as compared to cisplatin control (Table 4). Furthermore, 5HIAA concentration was also decreased in area postrema (*P* < 0.01). Combination 4 significantly (*P* < 0.001) decreased the upsurge of dopamine in the area postrema and 5HT in the brain stem and intestine (Table 4) as compared to cisplatin control. No significant changes were noted by Combination 4 on any of the neurotransmitter and their metabolites (Table 4).

## 4. Discussion

The current study is expedited to investigate the antiemetic effects of *Cannabis sativa* (*CS*), *Zingiber officinale* (*ZO)*, and *Bacopa monniera* (*BM*) alone or in combination against cisplatin induced vomiting in pigeon. *CS*, *ZO*, and *BM* extracts exhibited prominent antiemetic activity. Preparations containing the active phytochemical from *CS* were found effective against cisplatin induced vomiting (7 mg/kg) [58]. In continuation, our previous study reported *CS* antiemetic activity in pigeons where the hexane fraction proved to be very effective against cisplatin induced vomiting at the dose of 10 mg/kg single and twice daily dosing provided up to 58.5% (17 ± 3.4 episodes) and 65.6% (14.1 ± 2.9 episodes) protection, respectively [47]. In the current study, *CS*-HexFr 10 mg provided up to 62.2% (17 ± 2.7 episodes) protection against cisplatin induced vomiting (Table 1). The hexane fraction of *CS* extract contains all the nonpolar compounds and the active component-*Δ*^9^-THC. The *CS* major component *Δ*^9^-THC has been reported to have its clinical significance in the management of cisplatin induced vomiting [59]. CB_1_ receptors which are present presynaptically are involved in the mediation of antiemetic effect of THC, whose stimulation results in the inhibition of neurotransmitters which trigger the act of vomiting [60, 61]. The dose of 7 mg/kg was selected based on our previous study [45] which produced reliable vomiting response during the observation period and also not resulted in mortality.

*BM* belongs to family Scrophulariaceae and is present abundantly in Pakistan [62]. *BM* extracts are subjected to standardization in previous studies and our laboratory also did the standardization of plant extracts for quantification of bacosides by HPLC finger printing. The findings authenticate that the butanolic fraction contains the highest concentration of bacosides [43]. Clinical trials on bacosides for the management of memory enhancement establish the safety and tolerability of these phytochemicals and available currently in various herbal preparations alone or in combination. *BM* exhibit prominent antioxidant activity [63] and attenuate the dopamine receptor mediated hyperactivity [64]. The reports by our lab advocate that bacosides in a potent manner (~700 *μ*g/kg) suppress the vomiting induced by cisplatin up to 24 hours in pigeons [51] so it will be a good candidate to be used alone or in combination for the CIV management in clinics.

In this study, *BM*-MetFr 10 mg and *BM*-ButFr 5 mg attenuated cisplatin induced vomiting up to 35.6% (29 ± 4.3, *P* > 0.05) and 71.1% (13 ± 2.1) where *BM*-ButFr 5 mg provided more pronounced suppression (*P* < 0.001) as compared to *BM*-MetFr 10 mg and standard MCP. *BM* has proved to be better than the dopamine receptor antagonist – metoclopramide; which may reside in its ability to scavenge free radicals [63], suppression of dopaminergic, and serotonergic activity [43, 65].

*ZO* belonging to family *Zingiberaceae* having common name–Ginger. Ginger rhizome is cultivated throughout the Asian countries and is used as spice. The use of *ZO* for medicinal purposes is reported since long and is been added to Indian and Chinese pharmacopoeias. The acetone fraction which is reported to be gingerol rich fraction was screened for its antiemetic activity against cisplatin induced vomiting and provided up to 44.4% (25 ± 1.8) protection. The standardization of ginger extracts has the findings that up to 60 mg/g of gingerols are present in extract [66]. Postoperative nausea and vomiting is well managed by Ginger and the antiemetic results are almost equal to the antiemetic response by metoclopramide [67]. Our lab studies have reported the dose of 50 mg to be very effective in suppression of vomiting induced by cisplatin while the longer protection was observed with the dose of 25 mg [49]. There are so many reasons to support the antiemetic activity of ginger including the enhancement of gastroprokinetic activity, antiserotonergic effect [37], inhibitory action of substance P, and expression of NK_1_ receptors [68]. Our previous study [49] and current results (Table 1) supports the claim that ginger acetone fraction is having antiemetic activity.

Metoclopramide is dopamine receptor antagonist and also shares serotonin (5HT3) receptor blocking at high doses [69]; both the properties contribute in its antiemetic property. In the present study the dose of Metoclopramide used is based on a previous study [70]. Serotonin receptor blockers have showed intrinsic emetic activity in pigeons (Unpublished data) so the 5HT_3_ antagonist drugs were not used as standard antiemetic.

The multimechanisms behind the vomiting induced by cisplatin resulted in the use of antiemetics in combination and a single antiemetic fails for control both the phases of vomiting. The international guidelines also recommend the use of 5HT_3_ blockers, NK_1_ receptor antagonists, and dexamethasone in the management of both the phases of vomiting. Various combinations of plant extracts were tested in this study and one combination (No 4) was found to be synergistic and provided very nice remission of vomiting response (Table 1).

In continuation, the protection observed for *CS*-HexFr 10 mg alone was ~62.2% (Current study) and 55.45% in our previous published work [48] while for *BM*-ButFr 5 mg the protection observed was 71.1% (Current study) and 68.08% protection in our previous study [65]. Combination 2 was also found to be effective though less significant (*P* < 0.01) to combination 4 (Table 1).

In the current study, treatments with combination 4 do not changed basal neurotransmitters level and their metabolites any significantly. Furthermore, the decrease in the concentration of 5HIAA by MCP (30 mg) and combination 4 was observed at the brain stem (Table 2). The combination of *CS*-HexFr (10 mg) with *BM*-ButFr (5 mg) reduced 5HT and 5HIAA in the brain areas (AP and BS) and intestine (Table 3, *P* < 0.05–0.001). These findings are supportive for the antiemetic activity of Combination 4 for the 3^rd^ hour (at the acute vomiting response). Similar effect was also observed by metoclopramide. Combination of *CS*-HexFr 10 mg with *BM*-ButFr 5 mg suppressed the dopamine concentration in the brain area of AP as compared to cisplatin control while no significant dopaminergic suppression was seen in the BS and intestine (Table 4) at 18^th^ hour of cisplatin treatment. In continuation, Combination 4 (CS-HexFr 10 mg + *BM*-ButFr 5 mg) significantly (*P* < 0.001) reduced 5HT concentration at the level of BS and intestine (Table 4). The standard MCP (30 mg) also presented almost the same picture of neurotransmitter suppression in the brain area of AP, BS, and intestine. The antiserotonergic along with antidopaminergic effects noted of combination 4 in the current study is supporting the synergistic and prolongs protection provided against the vomiting induced by cisplatin in pigeons as compared to metoclopramide (Table 1).

## 5. Conclusions

In conclusion, the combination 4 provided a synergistic protection and our neurotransmitter quantification supports the involvement of antiserotonergic and antidopaminergic effects in an overlapping mode at the two different time points. At the acute time point (3^rd^ hour), dominantly the antiserotonergic effects were observed. Moreover, antidopaminergic and antiserotonergic effects were observed at the 18^th^ of cisplatin administration. These neurochemical findings advocate the promising antiemetic effect of combination 4 against cisplatin induced vomiting in pigeon. The combination may be useful alone or as adjunct in the management of cisplatin induced vomiting in clinics as *cannabis* preparations (Nabilone etc.) and preparations of *bacopa* (Bacomind®) are already available in the market and have safety and tolerability profile.

## Figures and Tables

**Figure 1:** Antiemetic effect of *CS* Hexane fraction (10 mg/kg), *BM* methanolic (10 mg/kg) and bacoside rich *n*-butanol fraction (5 mg/kg) and *ZO* acetone fraction (25 mg/kg) alone.

**Figure 2:** Antiemetic effect of combination of *CS* Hexane fraction (10 mg/kg), *BM* methanolic (10 mg/kg) and bacoside rich *n*-butanol fraction (5 mg/kg) and *ZO* acetone fraction (25 mg/kg).

**Figure 3:** Number of vomiting episodes observed after treatment with combination of *CS* Hexane fraction (10 mg/kg), *BM* methanolic (10 mg/kg) and bacoside rich *n*-butanol fraction (5 mg/kg) and *ZO* acetone fraction (25 mg/kg). Each column represents mean vomiting episodes after every 4 h ± S.E.M. ^∗^*P* < 0.05, ^∗∗^*P* < 0.01, ^∗∗∗^*P* < 0.001 as compared to control, two-way repeated measures ANOVA followed by Tukey's *post hoc* test.

**Table 1:** Effect of *CS* Hexane fraction (10 mg/kg), *BM* methanolic (10 mg/kg) and bacoside rich *n*-butanol fraction (5 mg/kg) and *ZO* acetone fraction (25 mg/kg) alone and in combinations on cisplatin induced *R+V* in pigeons.

Drug treatment	Dose & route	Pigeons n/vomited	*R + V* Mean ± sem	Latency (min) mean ± sem	Jerks Mean ± sem	Wt loss (%) mean ± sem
Saline+cisplatin	02 ml/kg i.m. +7 mg/kg i.v.	6/6	45 ± 1.9	66 ± 8.4	542 ± 84	15.5 ± 1.8
MCP+cisplatin	30 mg/kg i.m. +7 mg/kg i.v.	7/7	23.5 ± 0.3	248 ± 95	411 ± 112	10.8 ± 1.6
CS-HexFr+cisplatin	10 mg/kg i.m. +07 mg/kg i.v.	6/6	16.5 ± 2.7∗∗	258 ± 113	226 ± 84	7.5 ± 1.8
BM-MetFr+cisplatin	10 mg/kg i.m. +7 mg/kg iv	6/6	29 ± 4.3	243 ± 172	570 ± 138	8.9 ± 1.3
BM-ButFr + cisplatin	5 mg/kg i.m. +7 mg/kg iv	8/8	13 ± 2.1∗∗∗	137 ± 24	330 ± 95	9.1 ± 2.1∗
*ZO*-ActFr + cisplatin	25 mg/kg i.m. +07 mg/kg i.v.	8/8	25 ± 1.8	139 ± 21	223 ± 81	8.7 ± 1.4∗
(CS-HexFr + BM-MetFr) + cisplatin	(10+10 mg/kg i.m.) +7 mg/kg i.v.	6/6	30 ± 1.1	131 ± 16	672 ± 124	5.1 ± 2.5∗∗
(BM-ButFr + *ZO*-ActFr) + cisplatin	(5 + 25 mg/kg i.m.) +7 mg/kg i.v.	6/6	12 ± 0.4∗∗	69 ± 21	598 ± 194	9.6 ± 2.4
(*ZO*-ActFr + CS-HexFr) + cisplatin	(25+10 mg/kg i.m.) +7 mg/kg i.v.	7/7	19 ± 0.2∗	85 ± 12	415 ± 108	7.3 ± 1.9∗
(CS-HexFr + BM-ButFr) + cisplatin	(10+ 5 mg/kg i.m.) +7 mg/kg i.v.	6/5	05 ± 0.1∗∗∗	369 ± 123∗∗	99 ± 47	10.6 ± 1.7

Effect of *CS* Hexane fraction (CS-HexFr), *BM* methanolic fraction (BM-MetFr), bacoside rich *n*-butanol fraction (BM-ButFr), and *ZO* acetone fraction (*ZO*-ActFr) alone and in combinations on cisplatin induced vomiting and jerking during a 24 hr observation period. Standard metoclopramide (MCP; 30 mg/kg) is also shown. Values significantly different compared to cisplatin control are indicated as ∗*P* < 0.05, ∗∗*P* < 0.01, and ∗∗∗*P* < 0.001 (ANOVA followed by Tukey post hoc test). Combination 1 (CS-HexFr 10 mg + BM-MetFr 10 mg), Combination 2 (BM-ButFr 5 mg + *ZO*-ActFr 25 mg), Combination 3 (*ZO*-ActFr 25 mg + CS-HexFr 10 mg), and Combination 4 (CS-HexFr 10 mg + BM-ButFr 5 mg).

**Table 2:** Effect of metoclopramide (MCP) or combination (CS-HexFr 10 mg + BM-ButFr 5 mg) on basal level of neurotransmitters and their metabolites at the brain level of Area postrema (AP), Brain stem (BS), and intestine in pigeons.

Treatment	NA	DOPAC	DA	5HIAA	HVA	5HT
Area Postrema						
Saline	0.590 ± 0.011	0.470 ± 0.011	0.610 ± 0.139	0.175 ± 0.106	0.887 ± 0.083	0.059 ± 0.041
MCP 30 mg	0.031 ± 0.004	0.020 ± 0.010	0.032 ± 0.021	0.006 ± 0.011∗	0.120 ± 0.056∗	0.041 ± 0.002
(CS-HexFr 10 mg + BM-ButFr 5 mg)	1.491 ± 1.382	0.408 ± 0.276	0.225 ± 0.088	0.100 ± 0.044	1.096 ± 0.507	0.147 ± 0.095

Brain stem						
Saline	0.089 ± 0.021	0.063 ± 0.070	0.193 ± 0.067	0.071 ± 0.031	0.059 ± 0.020	0.012 ± 0.001
MCP 30 mg	0.120 ± 0.041	0.034 ± 0.004	0.050 ± 0.019	0.006 ± 0.010∗∗∗	0.073 ± 0.040	0.020 ± 0.020
(CS-HexFr 10 mg + BM-ButFr 5 mg)	0.160 ± 0.115	0.031 ± 0.000	0.428 ± 0.157	0.012 ± 0.003∗	0.104 ± 0.042	0.020 ± 0.006

Intestine						
Saline	0.187 ± 0.063	0.074 ± 0.010	0.087 ± 0.056	0.083 ± 0.049	0.071 ± 0.031	0.054 ± 0.013
MCP 30 mg	0.129 ± 0.047	0.063 ± 0.014	0.063 ± 0.021	0.012 ± 0.010	0.207 ± 0.012	0.071 ± 0.010
(CS-HexFr 10 mg + BM-ButFr 5 mg)	0.248 ± 0.040	0.123 ± 0.045	0.056 ± 0.001	0.029 ± 0.010	0.119 ± 0.115	0.063 ± 0.021

Effect of combination of CS-HexFr (10 mg) with BM-ButFr (5 mg) administered 30 minutes before saline administration, on the basal level of neurotransmitters and their metabolites (ng/mg tissue wet weight) at the brain level of AP and BS and Intestine in pigeons at *t* = 3 hr (*n* = 6 − 8). Standard MCP is also shown. Values significantly different compared to basal level are indicated as ∗*P* < 0.05, ∗∗*P* < 0.01, ∗∗∗*P* < 0.001 (ANOVA followed by Tukey post hoc analysis).

**Table 3:** Effect of standard metoclopramide (MCP), or combination of CS-HexFr (10 mg) with BM-ButFr (5 mg) on neurotransmitters and their metabolites at the brain level of area postrema (AP) and brain stem (BS) and intestine at 3^rd^ hour of cisplatin treatment.

Treatment	NA	Dopac	DA	5HIAA	HVA	5HT
Area Postrema						
Saline	0.701 ± 0.271	0.199 ± 0.010	0.763 ± 0.200	0.091 ± 0.040	0.900 ± 0.173	0.131 ± 0.050
Cisplatin	1.704 ± 1.401	0.408 ± 0.170	0.091 ± 0.270	0.379 ± 0.001#	0.607 ± 0.109	0.314 ± 0.110
MCP 30 mg	0.116 ± 0.078	0.142 ± 0.050	0.310 ± 0.137	0.026 ± 0.006∗∗	0.040 ± 0.021	0.030 ± 0.005∗
(CS-HexFr 10 mg + BM-ButFr 5 mg)	0.166 ± 0.139	0.192 ± 0.088	0.339 ± 0.144	0.046 ± 0.019∗∗	0.443 ± 0.181	0.048 ± 0.022∗

Brain stem						
Saline	0.117 ± 0.031	0.041 ± 0.020	0.260 ± 0.130	0.020 ± 0.010	0.070 ± 0.023	0.016 ± 0.001
Cisplatin	0.113 ± 0.040	0.185 ± 0.046	0.040 ± 0.010	0.057 ± 0.001###	0.032 ± 0.002	0.153 ± 0.011###
MCP 30 mg	0.041 ± 0.021	0.039 ± 0.003	0.013 ± 0.002	0.021 ± 0.001∗∗∗	0.023 ± 0.001	0.008 ± 0.000∗∗∗
(CS-HexFr 10 mg + BM-ButFr 5 mg)	0.089 ± 0.007	0.011 ± 0.001	0.119 ± 0.069	0.003 ± 0.002∗∗∗	0.018 ± 0.003	0.006 ± 0.002∗∗∗

Intestine						
Saline	0.416 ± 0.037	0.092 ± 0.010	0.129 ± 0.024	0.041 ± 0.000	0.107 ± 0.052	0.051 ± 0.001
Cisplatin	0.301 ± 0.047	0.024 ± 0.002	0.037 ± 0.004	0.304 ± 0.030###	0.043 ± 0.005	0.689 ± 0.104###
MCP 30 mg	0.109 ± 0.040∗	0.029 ± 0.001	0.246 ± 0.183	0.031 ± 0.006∗∗∗	0.067 ± 0.030	0.041 ± 0.005∗∗∗
(CS-HexFr 10 mg + BM-ButFr 5 mg)	0.266 ± 0.104	0.047 ± 0.275∗	0.399 ± 0.232	0.003 ± 0.001∗∗∗	0.004 ± 0.002	0.007 ± 0.006∗∗∗

Effect of combination of CS-HexFr (10 mg) with BM-ButFr (5 mg) administered 30 mins before cisplatin challenge, on the level of neurotransmitters and their metabolites (ng/mg tissue wet weight) at the brain level of AP and BS and Intestine of pigeons at *t* = 3 hr of cisplatin administration (*n* = 6 − 8). Standard MCP is also shown. Values significantly different compared to cisplatin control are indicated as ∗*P* < 0.05, ∗∗*P* < 0.01∗∗∗*P* < 0.001, while values significantly different compared to basal level are indicated as #*P* < 0.05, ###*P* < 0.001 (ANOVA followed by Tukey post hoc analysis).

**Table 4:** Effect of standard metoclopramide (MCP) or combination of CS-HexFr (10 mg) with BM-ButFr (5 mg) on neurotransmitters and their metabolites at the brain level of area postrema (AP) and brain stem (BS) and intestine at 18^th^ hour of cisplatin treatment.

Treatment	NA	Dopac	DA	5HIAA	HVA	5HT
Area Postrema						
Saline	0.507 ± 0.054	0.299 ± 0.129	0.520 ± 0.117	0.207 ± 0.020	0.863 ± 0.130	0.012 ± 0.011
Cisplatin	0.307 ± 0.056	0.021 ± 0.001	6.898 ± 1.300###	0.205 ± 0.048	0.584 ± 0.106	0.153 ± 0.040##
MCP 30 mg	0.250 ± 0.081	0.076 ± 0.041	0.125 ± 0.030∗∗∗	0.020 ± 0.010∗∗	0.383 ± 0.129	0.005 ± 0.002∗∗
(CS-HexFr 10 mg + BM-ButFr 5 mg)	0.471 ± 0.174	0.166 ± 0.066	0.504 ± 0.362∗∗∗	0.072 ± 0.012	1.388 ± 0.370	0.107 ± 0.029

Brain stem						
Saline	0.091 ± 0.004	0.083 ± 0.013	0.081 ± 0.041	0.193 ± 0.037	0.032 ± 0.020	0.010 ± 0.000
Cisplatin	0.090 ± 0.003	0.011 ± 0.001	0.192 ± 0.037	0.047 ± 0.002	0.008 ± 0.010	0.172 ± 0.001###
MCP 30 mg	0.012 ± 0.002	0.005 ± 0.001	0.021 ± 0.028	0.015 ± 0.003	0.097 ± 0.048	0.020 ± 0.001∗∗∗
(CS-HexFr 10 mg + BM-ButFr 5 mg)	0.277 ± 0.094∗∗∗	0.007 ± 0.002	0.074 ± 0.074	0.014 ± 0.002	0.022 ± 0.020	0.022 ± 0.004∗∗∗

Intestine						
Saline	0.317 ± 0.160	0.120 ± 0.060	0.193 ± 0.050	0.010 ± 0.001	0.041 ± 0.010	0.062 ± 0.013
Cisplatin	0.265 ± 0.029	0.013 ± 0.001	0.230 ± 0.031	0.340 ± 0.054	0.073 ± 0.005	0.506 ± 0.107###
MCP 30 mg	0.184 ± 0.059	0.021 ± 0.010	0.030 ± 0.010	0.031 ± 0.008	0.527 ± 0.435	0.037 ± 0.004∗∗∗
(CS-HexFr 10 mg + BM-ButFr 5 mg)	0.464 ± 0.060	0.001 ± 0.001	1.308 ± 0.240	0.020 ± 0.011	0.113 ± 0.112	0.047 ± 0.027∗∗∗

Effect of combination of CS-HexFr (10 mg) with *BM*-ButFr (5 mg) administered 30 mins before cisplatin challenge, on the level of neurotransmitters and their metabolites (ng/mg tissue wet weight) at the brain level of AP and BS and Intestine of pigeons at *t* = 18 hr of cisplatin administration (*n* = 6 − 8). Standard MCP is also shown. Values significantly different compared to cisplatin control are indicated as ∗∗*P* < 0.01∗∗∗*P* < 0.001, while values significantly different compared to basal level are indicated as ##*P* < 0.01 ###*P* < 0.001 (ANOVA followed by Tukey post hoc analysis).

## Data Availability

Data presented in the current manuscript belongs to the PhD work of Dr Ihsan Ullah and is not published anywhere. Data is available to researchers upon request.

## Abbreviations

CS: *Cannabis sativa*
BM: *Bacopa monniera*
ZO: *Zingiber officinale*
HPLC: High performance liquid chromatography
ECD: Electrochemical detector
5HT: 5-Hydroxy tryptamine
DA: Dopamine
HVA: Homovanillic acid
Dopac: Dihydroxy phenyl acetic acid
5HIAA: 5 Hydroxy indole acetic acid
CS-HexFr: *Cannabis sativa* (hexane fraction)
ZO-ActFr: *Zingiber officinale* (acetone fraction)
BM-ButFr: *Bacopa monniera* butanolic fraction
AP: Area Postrema
BS: Brain stem
HEC: Highly emetogenic chemotherapy
5HT3: 5 hydroxy tryptamine type 3
NK1: Neurokinin type 1
CIV: Chemotherapy induced vomiting
THC: Tetrahydrocannabinol
MCP: Metoclopramide
R+V: Retching+vomiting.
